The article "Genetic analysis of the CITED2 gene promoter in isolated and sporadic congenital ventricular septal defects" was published in 2021. Journal: J Cell Mol Med.

# Genetic analysis of the CITED2 gene promoter in isolated and sporadic congenital ventricular septal defects

**DOI:** 10.1111/jcmm.16218

**Published:** 2021-01-13

**Authors:** Si‐Qiang Zheng, Huan‐Xin Chen, Xiao‐Cheng Liu, Qin Yang, Guo‐Wei He

**Affiliations:** ^1^ Center for Basic Medical Research & Department of Cardiovascular Surgery TEDA International Cardiovascular Hospital Chinese Academy of Medical Sciences, & Graduate School of Peking Union Medical College Tianjin China; ^2^ The Institute of Cardiovascular Diseases Tianjin University Tianjin China; ^3^ Drug Research and Development Center Wannan Medical College Wuhu China; ^4^ Department of Surgery Oregon Health and Science University Portland OR USA

**Keywords:** congenital heart disease, gene, genetic, ventricular septal defect

## Abstract

Ventricular septal defect (VSD) is the most common congenital heart defect. Previous studies have reported genetic variations in the encoding region of CITED2 highly associated with cardiac malformation but the role of CITED2 gene promoter variations in VSD patients has not yet been explored. We investigated the variation of CITED2 gene promoter and its impacts on gene promoter activity in the DNA of paediatric VSD patients. A total of seven variations were identified by Sanger sequencing in the CITED2 gene promoter region in 400 subjects, including 200 isolated and sporadic VSD patients and 200 healthy controls. Using dual‐luciferase reporter assay, we found four of the 7 variations identified significantly decreased the transcriptional activity of the CITED2 gene promoter in HEK‐293 cells (*P* < .05). Further, a bioinformatic analysis with the JASPAR databases was performed and a cluster of putative binding sites for transcription factors was created or disrupted by these variations, leading to low expression of CITED2 protein and development of VSD. Our study for the first time demonstrates genetic variations in the CITED2 gene promoter in the Han Chinese population and the role of these variations in the development of VSD, providing new insights into the aetiology of CHD.

## 1 INTRODUCTION

Congenital heart disease (CHD) is the most prevalent inborn defect and the leading cause of infant mortality, affecting 1 out of 100 live and accounting for 30% of foetal losses.^1^, ^2^ Together with advances in diagnostic capacities, surgical techniques and catheter‐based treatments, these developments have resulted in a marked decrease in mortality from CHD during infancy and childhood.^3^ Nevertheless, after surgical repair, patients remain at high risk of ongoing disease burden including atrial arrhythmias, pulmonary hypertension and repeated need for surgery.^4^ These are resulting in significant increases in health services utilization during infancy, childhood, transition years, adulthood and in the geriatric age group.^4^ Besides, survival even in patients with simple lesions such as patent ductus arteriosus, atrial septal defect and ventricular septal defect (VSD) still lag the survival of the general population in the recent era.^5^ Therefore, a thorough understanding of the underlying causes of CHD will become ever more important to improve the prevention or treatment of patients with CHD.

The underlying aetiology of CHD remains poorly understood. Although it has long been thought that the development of CHD is substantially influenced by interaction and correlation between genetic and environmental factors, a large body of evidence indicates that genetic factors contribute to the majority of CHD.^6^, ^7^, ^8^ The promoter, regulatory region of DNA located 5′ upstream of a gene, plays an essential role in transcriptional regulation. It is well reported that DNA sequence variations in the gene promoter region may be associated with alterations in gene expression levels, putatively leading to disease.^9^, ^10^ Consequently, the analysis of promoter DNA sequence variations is important for the reason that it improves the diagnosis of disease‐causing DNA promoter variations and also expands our understanding of the role of transcriptional regulation in human disease.

CITED2 gene is a key member of the CITED family and is widely expressed in the embryo.^11^ Studies have identified CITED2 as a cardiac transcription factor (TF) that is essential to heart development. Lack of CITED2 in embryos can cause abnormal heart ring formation, as well as various cardiac malformations including atrial septal defect, VSD, transposition of great arteries, double outlet right ventricle, and tetralogy of Fallot.^12^ Among these CHDs, VSD is by far the most common CHD, with a birth prevalence of 2.62 per 1000 live births,^13^ whereas there are no studies focusing on CITED2 gene promoter region variations in patients with VSD. Thus, we hypothesized that variations in the CITED2 gene promoter may result in abnormal CITED2 gene expression, which may increase susceptibility to the formation of VSD. To test this hypothesis, we designed the present study to genetically analyse the DNA sequence of the CITED2 genes promoter region in VSD patients in comparison with the healthy controls and to functionally analyse the variations found in the promoter region.

## 2 MATERIALS AND METHODS

### 2.1 Study participants

This study enrolled 400 Han Chinese subjects. The study was approved by the Ethics Committee of TEDA International Cardiovascular Hospital and adhered to the tenets of the Declaration of Helsinki. Written informed consent was obtained from all subjects or the parents or guardians. From August 2018 to August 2019, 667 children with VSD underwent repair surgery at our hospital. Among those, 243 had isolated and sporadic VSD. Among those, 200 patients were matched with normal control (n = 200) who had the same ethnicity, gender and similar age were recruited in the study (Figure 1A). The control group was chosen from normal body checking or CHD screening programme at the hospital. All control subjects were confirmed either by clinical screening or plus echocardiography that confirmed no cardiac diseases.

**FIGURE 1:** A, Study flow diagram; B, Locations of the identified variations within the CITED2 gene promoter. The genetic variations are named according to the genomic DNA sequence of the human CITED2 gene (Genbank accession number NG_016169.1). The transcription start site is at the position of 5001 in the first exon

### 2.2 Sequence analysis

Genomic DNA was extracted from peripheral blood samples using the standard procedure. The sequences of the CITED2 promoter was taken from the Genbank database (https://www.ncbi.nlm.nih.gov/genbank). The accession number for CITED2 is NG_016169.1. Polymerase chain reaction (PCR) primers were designed to cover translational start sites as well as the potential 5′ promoter region of CITED2 in accordance with literature (Table 1).^14^ The promoter region of the human CITED2 gene (1418 bp, from −1197bp to + 220bp to the transcription start site) was generated by PCR and directly sequenced. The primers for Sanger sequencing were listed in Table 1. Subsequently, the above DNA sequences were compared with the wild‐type CITED2 gene promoter sequence.

**TABLE 1:** List of primers used in this study

Primers name	Sequences 5′‐3′	Location	Position
PCR primers			
CITED2‐F1	5′‐AAAGGAAGAGTCCCAGCCGT‐3′	3804	−1197
CITED2‐R1	5′‐TTTCTGCTCCGAAGACCGAG‐3′	5221	+220
Sequencing primers			
CITED2‐F1	5′‐AAAGGAAGAGTCCCAGCCGT‐3′	3804	−1197
CITED2‐F2	5′‐TAGCAGAAGCACACGTACCC‐3′	4195	−806
CITED2‐F3	5′‐CGAGTCCCCTTTTCCCGTAG‐3′	4579	−422
CITED2‐F4	5′‐GCTATCCCGGCAGGCTCTA‐3′	4687	−314
CITED2‐R1	5′‐TTTCTGCTCCGAAGACCGAG‐3′	5221	+220
Primers containing restriction sites			
CITED2‐KpnI^a^, ^b^	5′‐ (KpnI)‐**GG** GGTACCAAAGGAAGAGTCCCAGCCGT‐3′	3804	−1197
CITED2‐BglII^a^, ^b^	5′‐ (BglII)‐**CA** AGATCTTTTCTGCTCCGAAGACCGAG‐3′	5221	+220

Note

PCR primers are designed based on the genomic DNA sequence of the CITED2 gene (NG_016169.1). The transcription start site is at the position of 5001 (+1).

Abbreviations: F, forward; R, reverse.

^a^ Restriction sites are underlined.

^b^ Protective bases are presented in bold.

### 2.3 Plasmid constructs, cell culture and transfection

To functionally analyse the variations of CITED2 gene promoter, DNA fragments of wild‐type and variations in the CITED2 gene promoter region, containing the terminal restriction sites KpnI and BglII, were generated by PCR. Subsequently, by digestion with restriction enzymes, the wild‐type and variant fragments were subcloned into the KpnI/ BglII sites of the upstream of the firefly luciferase reporter gene plasmid (pGL3‐basic) to construct expression vectors that were validated by Sanger sequence analysis. The PCR primers with KpnI and BglII sites are shown in Table 1.

HEK‐293 cells were routinely cultured in MEM (Minimum Essential Medium, Gibco), supplemented with 10% FBS (Fetal Bovine Serum, Thermofisher), 100 units/ml penicillin and 100 μg/mL streptomycin at 37°C with 5% CO_2_. Cells were maintained and passaged when reaching 80% confluence, and then, 1 × 10^5^ cells were seeded into each well of a 96‐well plate 24 hours before transfection. Cells were transfected with the above‐constructed reporter plasmids, respectively, plus the expressing renilla luciferase reporter plasmid (pRL‐SV40) as an internal control to normalize the transfection efficiency in each well. An empty pGL3‐basic vector was used as a negative control.

### 2.4 Analysis with dual‐luciferase reporter assay

Firefly luciferase activity was measured 48 hours after transfection. Subsequently, cells were lysed and luciferase activities were measured by adding a luciferase substrate buffer using the dual‐luciferase reporter assay system according to the manufacturer's protocol. The promoter activities of the CITED2 gene promoter were normalized by the ratios of firefly luciferase activities to renilla luciferase activities. All experiments were performed three repeats independently.

### 2.5 Transcription factor binding sites prediction

For evaluating whether variations would disrupt or create the affinity of transcription factor binding sites (TFBS), putative TFBS for CITED2 gene variations were predicted online at JASPAR (http://jaspar.genereg.net/), an open‐access database for TF binding profiles.^15^, ^16^ The relative profile score threshold was set at 85%.

### 2.6 Statistical analysis

Results are represented as mean ± SEM for continuous variables and as the number for categorical variables. The quantitative data were compared by a standard Student's t test to calculate the statistical significance of the experimental results. Pearson's chi‐square was used in comparison with DNA sequence variation frequencies among VSD patients and healthy controls. Hardy‐Weinberg equilibrium test was carried out in both VSD and control groups to verify the effective risk of these genetic variations. All statistical analyses were performed using SPSS23.0 software. The significance level was set as *P* < .05.

## 3 RESULTS

### 3.1 The DNA sequence variations identified in VSD patients and healthy controls

A total of 400 subjects, including 200 VSD patients (99 males, 101 females, age ranging from 2 months to 14 years) and 200 sex‐ and age‐matched healthy controls (99 males, 101 females, age ranging from 5 months to 14 years), were recruited (Figure 1A).

There were 7 DNA variations detected by Sanger sequencing. The genotype distributions were in Hardy‐Weinberg equilibrium in both VSD group and control group (both *P* > .05).

Table 2 shows the details of these variations. Among those seven variations, four single‐nucleotide variations (SNV) [g.4078A>C (rs1165649373), g.4255C>T (rs1583069506), g.4698A>G (rs529363037) and g.4778G>T (rs9385859)], and one novel heterozygous variation (g.4933 C>A) were not found in controls. Further, the allele frequency of these five variations is less than 0.0001 in the NCBI dbSNP database and GnomAD database, and 2 of them [g.4778G>T (rs9385859) and g.4933C>A] have 0 allele frequency (Table 2). In addition, 2 of those 5 variations were discovered in two patients, respectively (Table 2). These five variations were further investigated for functional studies.

**TABLE 2:** Variations within the CITED2 gene promoters in VSD patients and controls

Variations	Position^b^	Genotypes	Controls^a^	VSD^a^	Allele frequency^c^	*P‐*value
g.4078A>C(rs1165649373)	−923 bp	AC	0	2	G = 0.00003	‐
g.4255C>T(rs1583069506)	−746 bp	CT	0	1	A = 0.0005	‐
g.4285T>G(rs12333191)	−716 bp	TG	31	38	C = 0.21789	.43
g.4357G>A(rs76757432)	−644 bp	GA	16	12	T = 0.09475	.56
g.4698A>G(rs529363037)	−303 bp	AG	0	1	C = 0.00010	‐
g.4778G>T(rs9385859)	−223 bp	GT	0	2	None	‐
g.4933C>A	−68 bp	CA	0	1	None	‐

Abbreviations: −, not applicable; VSD, ventricular septal defects.

^a^ Allele frequency in groups.

^b^ Variations are located upstream (−) to the transcription start site at the position of 5001 (+1) of CITED2 gene (NG_016169.1).

^c^ The allele frequency was obtained from NCBI dbSNP database and GnomAD database.

There were two variations that are common [g.4285T>G (rs12333191) and g.4357G>A (rs76757432)] in the control. These were excluded from further study.

### 3.2 Functional analysis of the variations by dual‐luciferase reporter assay

To further determine whether these variations in CITED2 gene promoter directly affect the activity of CITED2 promoter, we generated the different variant reporter plasmids based on the fragments of CITED2 promoter: empty pGL3 (negative control), pGL3‐WT (wild‐type CITED2 gene promoter), pGL3‐4078C, pGL3‐4255T, pGL3‐4698G, pGL3‐4778T, and pGL3‐4933A, respectively. These reporter gene assays were performed following the transfection of HEK‐293 cells.

As illustrated in Figure 2B, luciferase activity analysis showed that among the 5 genetic variations examined on the promoter activity, the reporter plasmids carrying 4 of those (4078C, 4698G, 4778T or 4933A) significantly decreased the luciferase expression, compared to the wild‐type (*P* < .05, Figure 2B). The rest one variation (4255T) did not have significant effect on the luciferase expression (*P* > .05, Figure 2B).

**FIGURE 2:** A, Sequencing chromatograms of the variations within the CITED2 gene promoter. For all the heterozygous variations [g.4078A>C (rs1165649373), g.4255C>T (rs1583069506), g.4698A>G (rs529363037), g.4778G>T (rs9385859) and g.4933 C>A], top panels show wild‐type and bottom panels show heterozygous DNA sequences, marked with arrows; B, Relative transcriptional activity of wild‐type and variant CITED2 gene promoters in HEK‐293 cells. Wild‐type and variant CITED2 gene promoters were cloned into reporter gene vector pGL3 and transfected into HEK‐293 cells. The transfected cells were collected, and dual‐luciferase activities were assayed. Empty vector pGL3‐basic was used as a negative control. The transcriptional activity of the wild‐type CITED2 gene promoter was designed as 100%. The relative activities of CITED2 gene promoters were calculated. Lanes 1, pGL3‐basic; WT, pGL3‐wild‐type; V1, pGL3‐4078A>C; V2, pGL3‐4255C>T; V3, pGL3‐4698A>G; V4, pGL‐4778G>T; V5, pGL3‐4933 C>A; *, *P* < .05; **, *P* < .01

### 3.3 Putative binding sites for TFs affected by genetic variations

The potential binding sites for TFs in the CITED2 gene promoter affected by variations were investigated by the online tool JASPAR core TF database.^15^, ^16^ The results indicated that variations may disrupt or create binding sites for TFs. The variation g.4078C may create binding sites for nuclear factor I‐C (NFIC), nuclear factor 1 X‐type (NFIX), and RHOXF1, and disrupt the binding sites for HOXB7, HOXC8, and Islet‐2. The analysis is summarized in Table 3. Among these TFBSs, ELK1, E2F1, E2F4 and SP1 have been reported as TFs that regulate the CITED2 expression.^17^, ^18^, ^19^, ^20^ Figure 3 is a schema illustrating the role of CITED2 gene promoter region variation, in combination with the analysis by the JASPAR database from the present study and previous studies.^17^, ^18^, ^19^, ^20^ The schema included those genes and pathways: CITED2, Isl1, Nkx2.5, Gata4, Tbx5, Lefty2, and Pitx2, HIF1α, TFAP2 family, Nodal pathway, and VEGF pathway (Figure 3).

**TABLE 3:** TFBS predicted by the JASPAR database and promoter activity affected by variations

Variations	Binding sites for transcription factors		Promoter activity
	Create	Disrupt	
g.4078A>C(rs1165649373)	NFIC,NFIX,RHOXF1	HOXB7,HOXC8,ISL2	↓
g.4255C>T(rs1583069506)	‐	REL,INSM1	No change
g.4698A>G(rs529363037)	TFAP2E	STAT3	↓
g.4778G>T(rs9385859)	ELF5,STAT3,ETS2,STAT1	E2F6,TFAP2A,TFDP1,ELK1	↓
g.4933C>A	‐	KLF15,SP1,KLF2,E2F6,KLF5	↓

Abbreviations: −, not applicable; TFBS, transcription factor binding sites.

**FIGURE 3:** Schema describes the role of CITED2 gene promoter region variations found from the present study and analysed by the JASPAR database in combination with previous studies. The low CITED2 promoter activity caused by the variations contributes to the low expression of CITED2. Consequently, the low expression of CITED2 may be directly involved in the development of VSD. In addition, it may decrease the activity of VSD‐relevant genes and pathways, such as Isl1, Nkx2.5, Gata4, Tbx5, Lefty2, Pitx2 and the Nodal pathway. The low expression of CITED2 may also lead to overexpression of certain cardiac‐related genes such as HIF1α and the VEGF pathway. Further, the low level of CITED2 protein may weaken the combination of CITED2 and ISL1, leading to VSD and may overexpress TFAP2 family, causing low expression of Pitx2 that hinders the formation of a normal heart and increases the risk of VSD

## 4 DISCUSSION

The present study for the first time in the isolated and sporadic VSD patients found that (a) there are five significant variations within the CITED2 gene promoter region; (b) four of these five variations (4778G, 4255C, 4078C or 4933A) caused cellular functional changes with a significant decrease in the CITED2 promoter activity by influencing TFBSs; and (c) the functional changes by these variations may affect a group of downstream genes and pathways and eventually cause VSD.

CITED2 is a main member of the conserved family of hypoxia‐inducible transcriptional co‐activators that are expressed throughout early embryogenesis and in embryonic stem cells of all vertebrates.^21^, ^22^ Studies have indicated that CITED2 plays a crucial role in expressional regulation and in early and later heart development.^11^, ^21^, ^23^, ^24^ A study found that CITED2 mutations in the coding region detected in VSD are associated with cardiac malformations.^25^ In particular, it was reported that cardiac‐specific deletion of CITED2 in mice caused myocardial compact layer thinning and VSD, as well as abnormal angiogenesis, revealing that CITED2 played an essential role in the growth and development of ventricular muscles and ventricular septal.^26^ As it is well known that the promoter is the crucial regulatory region of gene transcriptional regulation,^9^ based on the functions of CITED2 reported above, we hypothesized that variations within the CITED2 gene promoter region may disrupt the normal processes of gene activation, leading to disease. The cellular functional tests performed in this study have clearly demonstrated that the four variations in the CITED2 gene promoter region discovered in the present study significantly altered the transcriptional activity of CITED2. The experiments therefore support our hypothesis.

It is essential to know whether genetic variations create or disrupt a new TFBS in the understanding of disease‐causing gene regulatory mechanisms.^27^ In the present study, we performed bioinformatic analyses with the 4 discovered variations at the promoter region of the CITED2 gene that had cellular functional changes through the JASPAR database. We found that the variation of g.4778G>T may disrupt the potential binding sites for E2F1, a TF that participates in the development and differentiation of several tissues and in the regulation of glucose oxidation, oxidative metabolism, etc.^17^ It has been demonstrated by chromatin immunoprecipitation analysis that E2F1 proteins bond to the CITED2 gene promoter regulatory region and the expression increases CITED2 promoter activity.^17^ Further, g.4778G>T may also disrupt the potential binding sites for ELK‐1. A previous study on the CITED2 promoter showed that ELK‐1 protein bonded to the promoter of CITED2 and cooperatively increased HIF‐2α activity in the transcriptional activation of the CITED2 promoter.^18^

Another variation, g.4933 C>A may disrupt the binding site for SP1 that is critical for CITED2 expression. In fact, knocking down Sp1 diminished CITED2 promoter activity.^19^, ^20^

Considering the experimental results in the present study that these variations at the CITED2 promoter region down‐regulated the expression of CITED2 (Figure 2B), the above findings suggest that these variations may alter CITED2 gene transcription by disrupting or creating binding sites of the CITED2 promoter region for TFs, contributing to the low expression of CITED2. The consequence of this may be associated with the development of VSD.

Figure 3 is a schema that describes the role of CITED2 gene promoter region variations found from the present study and analysed by the JASPAR database in combination with previous studies. The low CITED2 promoter activity caused by the variations contributes to the low expression of CITED2, as shown in our study. Consequently, the low expression of CITED2 may be directly involved in the development of VSD.^12^, ^25^, ^28^ In addition, the low expression of CITED2 may decrease the activity of VSD‐relevant genes and pathways, such as Isl1, Nkx2.5, Gata4, Tbx5, Lefty2, Pitx2 and the Nodal pathway.^7^, ^26^, ^28^, ^29^ The low expression of CITED2 may also lead to overexpression of certain cardiac‐related genes such as HIF1α and the VEGF pathway.^12^, ^26^, ^28^, ^30^, ^31^ Further, the low level of CITED2 protein may weaken the combination of CITED2 and ISL1 leading to VSD leading to VSD,^26^, ^28^, ^29^ and may overexpress TFAP2 family,^12^, ^26^ causing low expression of Pitx2 that hinders the formation of a normal heart and increases the risk of VSD.^12^, ^26^

### 4.1 Limitations of the study

There are some limitations in this study. The sample size at this stage is relatively small. Further verification of CITED2 promoter variations in larger cohorts or in other populations is required. The validation in other syndromic types of VSD is also required. In addition, the degree of decreased transcriptional activity is rather small, and therefore, in vivo validation in animals needs to be performed in the future in order to confirm the role of these variations in the development of VSD or other CHDs.

## 5 CONCLUSION

In conclusion, the present study for the first time has identified genetic variations in the CITED2 gene promoter region in isolated and sporadic VSD patients in the Han Chinese population. Further, the variations have been demonstrated to significantly affect the CITED2 gene expression in cellular functional experiments. Bioinformatic analysis also demonstrated that these variations may be involved in the development of VSD. This study therefore provides new insights into the aetiology of CHDs and potential therapeutic strategy.

## CONFLICT OF INTEREST

The authors declare no conflict of interest with respect to the authorship and publication of this article.

## AUTHOR CONTRIBUTIONS

**Si‐Qiang Zheng:** Data curation (equal); Formal analysis (equal); Investigation (equal); Validation (equal); Writing‐original draft (equal). **Huan‐Xin Chen:** Conceptualization (equal); Data curation (equal); Formal analysis (equal); Validation (equal). **Xiao‐Cheng Liu:** Data curation (supporting); Resources (supporting). **Qin Yang:** Conceptualization (supporting); Resources (equal); Supervision (supporting). **Guo‐Wei He:** Conceptualization (lead); Data curation (equal); Formal analysis (lead); Funding acquisition (lead); Investigation (equal); Methodology (equal); Project administration (equal); Resources (equal); Supervision (lead); Validation (lead); Writing‐review & editing (lead).

## ETHICAL APPROVAL

The study was approved by the ethics committee of TEDA International Cardiovascular Hospital. Written informed consent was obtained from all the participants. All the procedures were performed under the tenets of the Declaration of Helsinki and relevant policies in China.

## Data Availability

The data that support the findings of this study are available from the corresponding author upon reasonable request.
